The article "Study on the Mechanism of Platelet-Released Clusterins Inducing Restenosis after Carotid Endarterectomy by Activating TLR3/NF-κb p65 Signaling Pathway" was retracted in 2023. Reason: concerns about the peer review.

# Study on the Mechanism of Platelet-Released Clusterins Inducing Restenosis after Carotid Endarterectomy by Activating TLR3/NF-*κ*b *p*65 Signaling Pathway

**DOI:** 10.1155/2022/7631126

**Published:** 2022-01-10

**Authors:** Qingyu Meng, Xichun Li, Mingyu Zhao, Shusen Lin, Xiangwen Yu, Guanglong Dong

**Affiliations:** Vascular Surgery Department, The Third Affiliated Hospital of Qiqihar Medical University, Qiqihar 161000, China

## Abstract

This study aimed to explore the role of clusterin released by platelet aggregation in restenosis after carotid endarterectomy. 35 patients who underwent carotid endarterectomy due to carotid artery stenosis were enrolled in this study. They were admitted to the Third Affiliated Hospital of Qiqihar Medical University from January 2018 to January 2019. All the patients were divided into two groups: the restenosis group and the nonrestenosis group, according to the follow-up results within 12 months. Peripheral blood was collected on the first day, 6 months, and 12 months after operation. The expression of CLU in serum of plasma and platelet culture medium was detected by an ELISA experiment. The vascular endothelial cells were cultured in vitro with 100 ng/mL of human recombinant CLU added to the medium. Cell proliferation, migration, and invasion were detected by CCK8, scratch, and Transwell invasion tests. The expression level of TLR3 and NF-*κ*b *p*65 proteins in cells was detected by western blot. TLR3 knockout plasmids in vascular endothelial cell lines were transfected. Cell proliferation and migration were detected by CCK8 and the scratch assay. The CLU content in peripheral blood plasma and supernatant of platelet culture medium was significantly higher in the restenosis group than that of the control group (*p*=0.003) 6 months after operation (*p*=0.047) and 12 months after operation (*p*=0.011). When CLU was added to vascular endothelial cell culture medium, the proliferation and migration were significantly enhanced. The TLR3/NF-*κ*b *p*65 protein expression level in cells also significantly increased. After the transfection of TLR3 knockout plasmids into vascular endothelial cell lines, CLU cannot promote the proliferation and migration of vascular endothelial cells. Platelet-released clusterin can induce vascular endothelial cell proliferation and migration by activating the TLR3/NF-kb *p*65 signaling pathway, leading to carotid artery restenosis after carotid endarterectomy.

## 1. Introduction

Carotid artery stenosis is one of the important factors leading to ischemic stroke [1]. The current global incidence is about 4.4%–7%, of which about 25%–30% of rigid artery stenosis is closely related to stroke [2]. Atherosclerosis in the neck is a common cause of this disease. The intima and plate of the lesion can be removed by carotid endarterectomy (CEA), a minimally invasive surgery, and the arterial anatomical passage can be restored. CEA has been proven to be effective in treating carotid artery stenosis and preventing ischemic stroke [3]. However, the treatment may cause a variety of complications, including surgery-related deaths, ischemic stroke, myocardial infarction, overperfusion syndrome, and postoperative restenosis [4, 5]. Yuichi et al. [6] found that the incidence of restenosis in patients with high platelet aggregation scores was significantly higher than that in patients with low scores, which could be an important and effective index to predict restenosis after CEA operation. Furthermore, studies have shown that platelet aggregation leads to the release of clusterin (CLU), which plays an important role in many cardiovascular and cerebrovascular diseases, such as cerebral amyloid angiopathy, atherosclerosis, and stenosis [7–9]. CLU has also been reported as a potential marker of restenosis and ischemia-reperfusion injury after carotid endarterectomy [10, 11]. However, there have been few studies on the mechanism of how it affects the prognosis of patients after carotid endarterectomy.

CLU is a highly conserved heterodimeric glycoprotein with a molecular weight of 75–80 kDa, consisting of two subunits connected by five disulfide bonds. It can be involved in many biological processes to play a wide range of functional characteristics [12, 13]. In recent years, many studies have shown that highly expressed CLU is closely related to cardiovascular diseases such as tissue degeneration, neurodegenerative diseases, malignant tumorigenesis, myocarditis, atherosclerosis, and so on [14, 15]. CLU expression cannot be detected in normal healthy blood vessels. But a high level of CLU in intimal smooth muscle cells can be detected in different stages of aortic injury and atherosclerosis development [16, 17]. It was found that CLU high expression may be related to the transition of vascular smooth muscle cells from proliferation to differentiation of contractile phenotype [18]. Secretory CLU mediates the formation of multicellular nodule aggregation in vascular smooth muscle cells and regulates smooth muscle cell migration, adhesion, and proliferation in vitro. All of the abovementioned findings suggest that the protein is involved in arterial wall remodeling [19]. This process is essential after carotid endarterectomy, suggesting that CLU plays a key role in the process of postoperative repair and remodeling. Nevertheless, the number of studies on serum CLU expression in patients with CEA is still small. There have been no experiments that detected the CLU of platelet release after operations. Therefore, this paper aimed to study the expression of clusterin in serum and the related mechanism of restenosis after CEA treatment, providing a new idea for carotid endarterectomy and prognosis.

In this study, peripheral blood was collected from patients with CEA on the first day, 6 months, and 12 months after the operation, and CLU expression level was detected by ELISA after peripheral blood plasma separation. The results showed that on the first day after surgery, the CLU expression level in the control group and the restenosis group was significantly increased, and after 6 and 12 months after operation, the CLU decreased significantly in the control group and the restenosis group. The CLU expression level in the restenosis group was still high, which was significantly higher than that in the control group, suggesting that the CLU of platelet origin may be CEA in postoperative restenosis. It may be used to indicate the prognosis of the patients, which was consistent with previous studies reported [11]. After angioplasty, CLU can be used as a predictor of restenosis in patients with coronary artery stenosis [20]. According to this, combined CLU plays an important role in many biological processes related to atherosclerosis and the cell cycle. We speculated that CLU can lead to vascular restenosis by affecting vascular endothelial cells.

## 2. Materials and Methods

### 2.1. Research Subjects

35 patients who underwent carotid endarterectomy due to carotid artery stenosis were enrolled in this study. They were admitted to the Department of Vascular Surgery, the Third Affiliated Hospital of Qiqihar Medical University, from January 2018 to January 2019. There were 21 males and 14 females, aged 48–69 years with an average age of (58.94 ± 1.01) years. According to the North American Symptomatic Carotid Endarterectomy Trial (NASCET), the degree of carotid artery stenosis was determined. The results showed that there were 3 patients with complete carotid artery occlusion, 9 patients with severe stenosis, and 10 patients with moderate stenosis. The inclusion criteria were as follows: (1) patients diagnosed as carotid artery stenosis with carotid stenosis using carotid ultrasound, transcarotid magnetic resonance angiography, computed tomographic angiography (CTA), and/or digital subtraction angiography (DSA); (2) patients operated by the same group of CEA physicians through a jugular incision, intraoperative foreign body implantation; and (3) patients without a history of severe neck trauma, neck tumor, or radiotherapy. The exclusion criteria were as follows: (1) patients who could not be followed up with ultrasound and blood collection; and (2) patients who were treated with antiplatelet agents during postoperative recovery. All included patients received a 1-year follow-up visit. Peripheral blood was taken at 1 day, 6 months, and 12 months after surgery and carotid ultrasound were performed. The patients were divided into two groups: the restenosis group and the nonrestenosis group according to the return visit. The restenosis group included patients whose lumen diameter was reduced by more than 50% (area decreased by 75%) based on a standard contraction peak velocity of >1.25 m/s or a contraction peak ratio of 2.0. This study has been approved by the Ethics Committee of the Third Affiliated Hospital of Qiqihar Medical University. All patients have been informed of the purpose and protocol of the experiment before drawing blood and have signed the informed consent.

### 2.2. Platelet Separation and Culture

2 ml of peripheral venous blood was extracted from all subjects by a sodium citrate anticoagulant tube, which was processed according to the human peripheral blood platelet separation solution kit (P6390, SolarBio). After the whole blood was diluted with an equal volume of PBS, two times the volume of the separation solution was added and centrifuged at 250 g at room temperature for 15 min to delimit. The top platelet-rich plasma layer was absorbed into the centrifuge tube, and 10 ml of PBS was added and centrifuged at 500 g for 20 min for washing. DMEM was added to the precipitate after centrifugation, and its concentration was adjusted to 2 × 106 pieces/mL. Then, 250 µg/ml fibrinogen was added to the medium. After 24 h, the unattached cells were washed off with PBS, and a fresh medium was added. After 24 h of continuous culture, 1000 g of supernatant of the cells was collected and centrifuged for 5 min and stored in a refrigerator at −80°C for later use.

### 2.3. CLU Expression Level Test

2 ml of peripheral venous blood was extracted from all subjects by a sodium citrate anticoagulant tube. The sample was set aside at room temperature for 30 min, then centrifuged to separate the serum, and stored in the refrigerator at −80°C. The concentration of clusterin in peripheral blood and platelet culture supernatant was determined by enzyme-linked immunosorbent assay (ELISA) according to the instructions of the CLU kit (ab174447, Abcam).

### 2.4. Cell Culture

HMEC-1 cell lines of vascular endothelial cells were purchased from ATCC cell banks, which were cultivated in the endothelial media (1001, ScienCell) with 5% fetal bovine serum (04-007-1 A, BI) and 1% endothelial growth factor (CYT-217, ProSpec). Then, the cells were placed in a 37°C thermostat incubator containing 95% air and 5% CO2, which were used when the density increased to 90%. After that, the cells were divided into the control group and the treatment group. 100 ng/mL human serum purified CLU (ab242207, Abcam) was added to the cell culture medium of the treatment group. After coculture for 24–48 h, the cells were grown to a suitable concentration for use.

### 2.5. CCK Experiment

HMEC-1 cells in the logarithmic growth phase were digested by trypsin (C0202, Biyuntian). The cell suspension (5 × 10^4^/mL) was prepared and added to a 96-well plate according to 100 *μ*L/well. The cells were placed in an incubator at 37°C until the cells adhered to the wall and covered the bottom of the well. At the same time, 10 *μ*l CCK8 solution was added to each hole. After mixing and incubating in the incubator for 2 hours, the absorption value was measured at 450 nm wavelength by an enzyme labeling instrument. The cell proliferation was calculated according to the formula.

### 2.6. Transwell Migration Experiment

1 × 10^5^ HMEC-1 cells were evenly inoculated into the Transwell chamber (3428, Corning). 500 *μ*l DMEM of 15% fetal bovine serum was added to the lower chamber, and cultivated in the incubator at 37°C with 5% CO_2_ for 24 h. The cells in the upper layer of the filter membrane were wiped off with a cotton swab, and the upper chamber was placed in methanol for fixation for 5 min. The cells were stained with Giemsa dye for 15 min. Five different fields of vision were selected under a 100x light microscope, and the number of membrane cells was penetrated by this technique.

The cells were placed in an incubator at 37°C overnight to cover the whole orifice plate. Straight scratches were drawn with the sterilizer head perpendicular to the bottom of the orifice plate. Then, it was rinsed with PBS buffer 3 times to wash off the scratched cells. The serum-free medium was added and put into an incubator at 37°C. After 0, 6, 12, and 24 hours of culture, the appropriate location was photographed, and the cell migration ability was analyzed.

### 2.7. Transwell Invasion Test

After diluting the Matrigel adhesive (354230, Corning) at a ratio of 1 : 10, the coating was placed at the bottom of the upper chamber of the Transwell orifice plate (3422, Corning). Then, it was incubated at 37°C for 30 min to polymerize the Matrigel into a gel. The cells were digested with trypsin, resuspended with serum-free medium containing BSA and adjusted to 5 × 10^5^/mL cell suspension, and 100 *μ*l of cells were added into the Transwell chamber. 600 *μ*l of culture medium with 20% FBS was added to the lower chamber of the orifice plate and removed out of the chamber after cultivating for 12–48 h. After being fixed with methanol for 30 min, the cells were stained with 0.1% crystal violet for 20 min. Five fields were randomly selected under a 400x microscope for observation and counting.

### 2.8. Western Blot Test

The proper amount of lysate (R0020, Solarbio) was added to the cells of the control and treatment groups to extract the total proteins by centrifugation after cell lysis. The BCA kit (P0012S, Biyuntian) was used to detect the protein concentration. The total proteins were gelled in an SDS-PAGE gel, and the target protein was transferred to the PVDF membrane by the semiwet transfer method. TLR3 (1 : 2000, ab62566, Abcam), NF-kBP65 (1 : 2000, ab16502, Abcam), and GAPDH (1 : 5000, ab8245, Abcam) antibody dilutions were added after BSA closure, which was kept at 4°C overnight. Then, it was washed with 0.1% PBST 3 times. The corresponding sheep anti-rabbit/mouse immune second antibody (1 : 2000, SA00001-1/2, Proteintech) was added to incubate for 1 h at room temperature. ECL chemiluminescence solution (P0018FS, Biyuntian) was added after washing 3 times. The image was developed, fixed, and recorded in a dark room, and the processing software ImageJ 1.52 was used for analysis.

http://www.ptgcn.com/Products/HRP-conjugated-Affinipure-Goat-Anti-Mouse-IgG-H-L--secondary-antibody.htm.

### 2.9. TLR3 Plasmid Transfection

TLR3 knockout and no-load plasmids were purchased from Shanghai Jima Pharmaceutical Company. When the cell density increased to 80–90%, the transfection reagent Lipofectamine 2000 (11668500, Invitrogen) was used to transfer the empty plasmid and TLR3 knockout plasmid of vascular endothelial cells. The transfection efficiency was determined by a fluorescence microscope. The total cell proteins were collected and placed in the refrigerator at −80°C.

### 2.10. Statistics and Analysis of Data

The software SPSS 23.0 was used for statistics and analysis of all the data. Measurement data was presented in the form of mean ± standard deviation ($\bar{x}\pm s$). A Chi-square test was used to detect whether there were differences in general conditions in patients with carotid artery stenosis in the nonrestenosis group and the restenosis group. The expression level of clusterin in peripheral blood and platelet culture supernatant was also analyzed by the Chi-square test, and the *t* test was used for paired samples and comparisons between groups. *p* < 0.05 was statistically significant.

## 3. Results

### 3.1. The Expression of Clusterin in the Serum of Peripheral Blood and Platelet Culture in the Patients of the Restenosis Group Increased Significantly

There were a total of 24 patients in the nonrestenosis group, including 16 males and 8 females. There were 11 patients in the restenosis group, including 5 males and 6 females, with an average restenosis time of 7.8 ± 2.5 months. The smoking rate in the restenosis group was significantly higher than that in the nonrestenosis group. However, there was no significant difference in age, sex, degree of arteriosclerosis, drinking rate, past medical history, and other diseases (Table 1). The ELISA method was used to detect the CLU concentrations in the restenosis and control groups. The results showed that at 6 months (82.00 ± 6.63 ng/ml *vs.* 56.92 ± 7.62 ng/ml, *p*=0.047) and 12 months (61.09 ± 6.94 ng/ml *vs*. 37.75 ± 4.93 ng/ml, *p*=0.011), the CLU expression level in the peripheral blood of the restenosis group was significantly increased (Figure 1). The CLU content in platelet culture medium supernatant of the restenosis group was significantly higher than that of the control group (105.2 ± 15.2 ng/ml *vs*. 49.73 ± 6.23 ng/ml, *p*=0.003).

### 3.2. Platelet-Derived Clusterins Can Lead to Increased Proliferation and Migration of Vascular Endothelial Cells

CCK8 and the scratch assay were used after adding 100 ng/mL of human recombinant CLU to the vascular endothelial cell culture medium. The results showed that CLU could promote the proliferation and migration of vascular endothelial cells (Figure 2(a)), while the Transwell invasion test showed no significant change in cell invasion ability (Figure 2(d)).

### 3.3. Platelet-Derived Clusterins Can Promote the TLR3/NF-kb Pathway Activation in Vascular Endothelial Cells

The western blot results showed that the expression of NF-kb *p*65 protein in TLR3 and downstream increased significantly after the addition of human recombinant CLU to vascular endothelial cell lines. The results suggest that clusterin may promote the proliferation and migration of vascular endothelial cells by activating the TLR3/NF-kb pathway (Figure 3).

Western blot test for the total TLR3 and *p*65 protein expression in the recombinant CLU group and the control group.

### 3.4. The Increased Capacity of Proliferation and Migration in Endothelial Cells Depends on the Agglutinin-Dependent Activation of TLR3 Signaling Pathways

The results showed that the deletion of TLR3 expression could significantly inhibit the proliferation (Figure 4(a)) and migration of vascular endothelial cells (Figures 4(b)-4(c)). Moreover, knockdown of TLR3 in endothelial cells can eliminate the CLU's role in promoting the proliferation and migration of vascular endothelial cells, suggesting that clusterin's role in the biological function of vascular endothelial cells depends on the activation of TLR3 signaling pathways.

## 4. Discussion

At present, it is considered that the most important factor in the pathogenesis of cerebral apoplexy is the lumen stenosis caused by carotid atherosclerosis. Cerebral apoplexy is characterized by high incidence and high mortality, which is a common cause of death in China. A large number of multicenter clinical studies have confirmed that carotid endarterectomy is the most mature method to prevent cerebral apoplexy in internal carotid atherosclerotic diseases, with great and long-lasting benefits [21]. However, there have been studies reporting that after CEA, there is a risk of postoperative restenosis. Patients with restenosis will have a significantly increased risk in the incidence of terminal stroke. Generally, re-intervention is needed in this situation. Therefore, restenosis after CEA greatly limits the benefits of CEA. To overcome this problem, recent studies have suggested that lifestyle, blood pressure, and blood glucose can be controlled. Antiplatelet agents, statins, or lipid-lowering agents such as ezetimibe can be used. The above methods may be beneficial for asymptomatic patients with carotid stenosis who require invasive revascular surgery [22, 23]. However, this management strategy does not solve the problem of postoperative restenosis, so this paper studied the mechanism of vascular restenosis to provide new targets and ideas for the prevention and treatment of restenosis after carotid endarterectomy.

There was a previous retrospective study, which divided 36 patients into high-rated and low-rated groups based on postoperative platelet aggregation scores. The authors found that the incidence of restenosis in the high-rated platelet aggregation group was significantly higher than that in the low-rated group, 50.0% and 13.6%, respectively [6]. Although the experiment included only 36 postoperative patients with CEA and may have had some bias in excluding patients who did not take aspirin, platelets can play an important role in the development of carotid artery restenosis. On this basis, there was another article that reported that platelets in cerebral vessels can promote CLU expression and thus mediate *β*-amyloid precipitation to cause amyloid angiopathy [7]. Therefore, we hypothesized that restenosis after CEA may be related to CLU resulting from platelet aggregation in the carotid arteries.

Vascular restenosis is mainly caused by excessive proliferation of vascular endothelium and smooth muscle [24]. Among them, vascular endothelial cells are the main ones that form the vascular wall. In addition, vascular endothelial cells can secrete a variety of cytokines, regulate the shape of smooth muscle cells around them, relax, and mediate vascular reconstruction. It plays an important role in atherosclerosis, diabetic vascular disease, restenosis, and vascular remodeling after coronary intervention [25]. As a result, we used the vascular endothelial cell line HMEC-1 for in vitro culture. We observed the changes of cell proliferation, migration, and invasion ability by adding human recombinant CLU with plasma concentration into the supernatant of vascular endothelial cells. The results showed that CLU activated the TLR3/NF-*κ*B signaling pathway and significantly enhanced cell proliferation and migration, and the process was found to be TLR3-dependent by the recovery experiment.

## 5. Conclusion

Existing studies have shown that high expression in TLR3 glomerular endothelial cells can lead to increased secretion of various cytokines, including IL-6, CX3CL1, and VCAM-1 [26–28]. However, this study has some limitations. The downstream target molecules mediated by the TLR3/NF-*κ*B signaling pathway have not been further analyzed, and the conclusions have not been verified in animal models, which will be further discussed in future studies. This study explored the level of clusterins released from peripheral blood plasma and platelets in patients with postoperative restenosis and nonrestenosis after CEA and examined the effects of CLU on the biological function of vascular endothelial cells. We found that platelet-derived clusterins can lead to vascular endothelial cell proliferation and migration by activating the TLR3/NF-kb *p*65 signaling pathway, which may lead to carotid artery restenosis after CEA. Therefore, it may lead to carotid artery restenosis after CEA, which lays the foundation for CLU to become a prognostic predictor and intervention target for patients after carotid endarterectomy.

In conclusion, platelet-released clusterin can induce vascular endothelial cell proliferation and migration by activating the TLR3/NF-kb *p*65 signaling pathway, leading to carotid artery restenosis after carotid endarterectomy.

## Figures and Tables

**Figure 1:** Expression level of clusterin in serum of peripheral blood and platelet culture in the control and restenosis groups. (a) Peripheral blood was collected on the first day (POD1), 6 months (POM6), and 12 months (POM12) after operation in the control and restenosis groups. The expression level of serum clusterin were detected by ELISA. (b) ELISA was also used to detect the expression of clusterin in platelet culture supernatant in the nonrestenosis and restenosis groups.

**Figure 2:** Platelet-derived clusterins can lead to increased proliferation and migration of vascular endothelial cells. (a) Experimental results of CCK8 in 100 ng/mL of the human recombinant CLU group and the control group in vascular endothelial cell medium. (b) Statistical results of Transwell migration experiments. (c) Transwell migration assay for cell migration between the recombinant CLU group and the control group. (d) Transwell invasion test for the invasion ability of the recombinant CLU group and the control group. ^*∗*^*p* < 0.05; ns, there was no statistical difference.

**Figure 3:** Platelet-derived clusterins can promote the TLR3/NF-kb pathway activation in vascular endothelial cells.

**Figure 4:** Increased capacity of endothelial cells to proliferate and migrate depends on the agglutinin-dependent activation of TLR3 signaling pathways. (a) CCK8 test for the cell proliferation of the control group, the TLR3 knockout group, the recombinant CLU group, and the TLR3 knockout + recombinant CLU group. (b–c). Transwell migration test for the cell migration of the control group, the TLR3 knockout group, recombinant CLU group, and the TLR3 knockout + recombinant CLU group. ^*∗*^*p* < 0.05; ns, there was no statistical difference.

**Table 1:** General situation of patients with carotid artery stenosis in the nonrestenosis and restenosis groups.

	Nonrestenosis group (*n*=24)	Restenosis group (*n*=11)	*p* value
Gender (M/F)	16/8	5/6	0.283
Age	58.79 ± 1.24	59.27 ± 1.81	0.829
*Level of carotid artery stenosis*			
Moderate stenosis	9	5	
Severe stenosis	11	3	
Complete occlusion	4	3	0.551
Smoking	10 (41.7%)	5 (45.4%)	0.833
Drinking	7 (29.2%)	5 (45.4%)	0.346
Hypertension	8 (33.3%)	8 (72.7%)	0.029^*∗*^

## Data Availability

The datasets used and/or analyzed during the current study are available from the corresponding author on reasonable request.
